The article "Intracranial Osteoma: Unusual Etiology of Chronic Daily Headaches" was retracted in 2024. Reasons: false authorship; unreliable results or conclusions; no approval from an author; concerns about the authorship.

# Intracranial Osteoma: Unusual Etiology of Chronic Daily Headaches

**DOI:** 10.7759/cureus.21488

**Published:** 2022-01-22

**Authors:** Nasser S Aldandan, Amal N Al Mutairi, Talal H Almutairi, Ayman M Aboalam, Turki A Saad, Abdullah K Alshebili, Mohammad K Almihmadi, Abdullah E Alzeer, Mohammed A Alhamyani, Alya M Alhazmi, Mariam H Fardous, Ghada A Alharbi, Maryam F Oraif, Bashaer O Abdu, Faisal Al-Hawaj

**Affiliations:** 1 Medicine, King Faisal University, Hofuf, SAU; 2 Medicine, Qassim University, Al-Qassim, SAU; 3 Medicine, King Saud bin Abdulaziz University for Health Sciences, Riyadh, SAU; 4 Medicine, King Khalid University, Abha, SAU; 5 Medicine, Medical University of Lodz, Łódź, POL; 6 Medicine, University of Debrecen, Debrecen, HUN; 7 Medicine, Taif University, Ta'if, SAU; 8 Medicine, Umm Al-Qura University, Mecca, SAU; 9 Medicine, King Saud Bin Abdulaziz University for Health Sciences, Riyadh, SAU; 10 Medicine, Dar Al Uloom University, Riyadh, SAU; 11 Medicine, Ibn Sina National College for Medical Studies, Jeddah, SAU; 12 Medicine, Imam Abdulrahman Bin Faisal University, Dammam, SAU

**Keywords:** calcification, case report, computed tomography, osteoma, headache

## Abstract

Headache is one of the most frequent complaints in the outpatient department. The types of headaches can be broadly classified into primary and secondary. The primary headaches have benign intrinsic causes and include tension, migraine, and cluster headaches. A detailed history and appropriate physical examination are essential in assessing patients with headaches.

We present the case of a 33-year-old woman who presented to our primary care clinic with three days history of worsening frontal headache. She had been experiencing this headache daily for the last three months; however, the current episode is more severe. The headache episode was not associated with fever, neck stiffness, or loss of consciousness. She often became nauseated with the headache. There was no history of weakness, numbness, or visual disturbances with the headache. There was no family history of migraine headaches. On examination, no focal neurological deficit was noted. The head CT scan showed the presence of two highly hyperdense foci in the frontotemporal region, one of them was related to the dura. Such foci were not causing midline shift or brain edema. The preliminary diagnosis was calcified meningioma. Surgical excision of the lesions was planned. The patient underwent right craniotomy under general anesthesia. The two osseous lesions were observed and successfully resected. Histopathological examination of the lesions was consistent with osteoma. Intracranial osteoma is a very rare benign neoplasm of the mature bone tissue. The typical clinical manifestation of intracranial osteoma is a chronic headache. Head CT shows a well-defined, hyperdense structure. However, this is often mistaken as calcified meningioma.

## Introduction

Headache is one of the most frequent complaints in the outpatient department. The types of headaches can be broadly classified into primary and secondary. The primary headaches have benign intrinsic causes and include tension, migraine, and cluster headaches [1]. A detailed history and appropriate physical examination are essential in the assessment of patients with headaches. Since the vast majority of headache episodes are benign, the key role of treating physicians is to identify the patients at risk for the serious cause of their headaches. Misdiagnosis of headache types may result in detrimental outcomes, including permanent neurological damage, vision loss, and death. Further, chronic daily headaches are prevalent worldwide, affecting up to 5% of the adult population with female predilection [2]. The chronic daily headache can be a cause of reduction in quality of life and excessive economic cost to the society [3]. Here, we present the case of a young woman with a chronic headache due to dural osteoma, an unusual etiology of chronic headache.

## Case presentation

A 33-year-old woman presented to our primary care clinic with three days history of worsening frontal headache. She had been experiencing this headache daily for the last three months; however, the current episode was more severe. She described the headache as pressure across her head. The headache was bilateral and was not radiating. She reported not having any warning signs before the headache. The headache was not related to the menstrual cycle or her diet. However, the headache worsened when she was stressed. It was not awakening her from her sleep. She scored it as 6 out of 10 on the severity scale. The headache episode was not associated with fever, neck stiffness, or loss of consciousness. However, she often became nauseated with the headache. There was no history of weakness, numbness, or visual disturbances with the headache. She reported that the headache has significantly affected her quality of life. The past medical history was remarkable for diabetes mellitus that was well-controlled with metformin 1000 mg. She was not a smoker and never drank alcohol. There was no family history of migraine headaches. She worked as a school teacher and found her job very stressful.

On examination, she was fully oriented to time, place, and person. No focal neurological deficit was noted. The tone and power were normal in both the upper and lower extremities. The coordination was intact, and the Babinski sign was negative. All examination findings were unremarkable. The patient was referred to undergo a head CT scan to rule out any space-occupying lesion, considering the chronicity of the pain. The scan showed the presence of two highly hyperdense foci in the frontotemporal region, one of them was related to the dura. Such foci were not causing midline shift or brain edema (Figure 1). The preliminary diagnosis was calcified meningioma. Subsequently, brain MRI re-demonstrated these foci with susceptibility artifact in keeping with calcified structures (Figure 2). No other abnormalities were observed.

**Figure 1:** Head CT showing two highly dense lesions (arrow) with no surrounding edema or mass effect.

**Figure 2:** T2-weighted MRI showing susceptibility artifact (arrow) in keeping with the calcified lesions.

The findings were discussed with the patient, and she was referred to the neurosurgery team for further management. Surgical excision of the lesions was planned. The patient underwent right craniotomy under general anesthesia. The two osseous lesions were observed. One lesion was attached to the dura mater, while the other had no dural attachment. Both lesions were successfully removed. Histopathological examination of the lesions consisted of mature bone (Figure 3). The patient had an uneventful recovery. She was discharged after seven days of hospitalization. In the follow-up visit, she reported a resolution of her chronic headache.

**Figure 3:** Histopathological image showing mature bone tissue in keeping with osteoma.

## Discussion

We reported the case of dural osteoma as a cause of chronic daily headaches. Osteoma is a benign tumor of mature bone tissue. In the head and neck region, osteoma more frequently involves the sinuses with attachment to the inner and outer tables of the skull bones [4]. However, it is very rare for osteoma to develop in the brain parenchyma with no attachment to the skull bones [5]. In the present case, there were two osteomas, with one of them having no skull bone involvement.

A limited number of cases have been reported about intracranial osteoma. It is reported to be more prevalent among women with a mean age of 42 years [4]. As in the present case, the most common presentation of intracranial osteoma is a headache. However, seizures and alterations in mental status may develop. The exact pathogenesis of intracranial osteoma is incompletely understood [6]. It has been suggested that intracranial osteoma may develop because of the presence of osteogenic activity of the dura, or it may arise from primitive mesenchymal cells [4].

Neuroimaging studies are essential to make the diagnosis. The presence of well-defined lesions with high attenuation on CT scans is the characteristic feature of osteoma. However, misdiagnosis of osteoma as calcified meningioma can occur, as in the present case. In fact, most of the reported intracranial osteoma in the literature were initially diagnosed as meningioma, and the correct diagnosis was made after the histopathological examination, which is the gold standard for diagnosis [6]. However, in the histopathological examination of intracranial osteoma, the lesion appears as a mature osseous lesion. Therefore, craniotomy for resection of intracranial osteoma is the treatment of choice with a good outcome [4].

## Conclusions

Intracranial osteoma is a rare, benign neoplasm of the mature bone tissue. The typical clinical manifestation of intracranial osteoma is a chronic headache. Head CT shows a well-defined, hyperdense structure; however, this is often mistaken as calcified meningioma. Hence, radiologists should always remember intracranial osteoma as a differential diagnosis of calcified meningioma. A craniotomy is considered a safe and effective treatment for intracranial osteoma.
